# A New Optimal Diagnosis System for Coronavirus (COVID-19) Diagnosis Based on Archimedes Optimization Algorithm on Chest X-Ray Images

**DOI:** 10.1155/2021/7788491

**Published:** 2021-08-21

**Authors:** Liping Chen, Tahereh Rezaei

**Affiliations:** ^1^College of Computer, Weinan Normal University, Weinan, Shaanxi, China; ^2^Neuroscience Research Center, Shiraz, Iran

## Abstract

The new coronavirus, COVID-19, has affected people all over the world. Coronaviruses are a large group of viruses that can infect animals and humans and cause respiratory distress; these discomforts may be as mild as a cold or as severe as pneumonia. Correct detection of this disease can help to avoid its spreading increasingly. In this paper, a new CAD-based approach is suggested for the optimal diagnosis of this disease from chest X-ray images. The proposed method starts with a min-max normalization to scale all data into a normal scale, and then, histogram equalization is performed to improve the quality of the image before main processing. Afterward, 18 different features are extracted from the image. To decrease the method difficulty, the minimum features are selected based on a metaheuristic called Archimedes optimization algorithm (AOA). The model is then implemented on three datasets, and its results are compared with four other state-of-the-art methods. The final results indicated that the proposed method with 86% accuracy and 96% precision has the highest balance between accuracy and reliability with the compared methods as a diagnostic system for COVID-19.

## 1. Introduction

Coronaviruses are a large family of viruses that can infect animals and humans. Many of the known coronaviruses have caused a range of respiratory infections in humans, ranging from the common cold to more severe illnesses such as Middle East Respiratory Syndrome (MERS) and Severe Acute Respiratory Syndrome (SARS). The newly discovered coronavirus is the cause of COVID-19 disease. The emerging virus and its disease were unknown before the recent outbreak.

COVID-19 is a new infectious disease that first broke out in December 2019 in Wuhan Province, China.

The disease later spread to other countries in Asia, Europe (mainly Italy, Spain, France, and the United Kingdom), Africa, and the United States (mainly the United States). The COVID-19 disease is highly transmissible. According to the World Health Organization (WHO), as of Apr 14, 2021, there are 13,804,929 cases of infection and 2,972,662 deaths. However, these statistics are exponentially increasing. From the outset, the World Emergency Committee stressed the need for prompt diagnosis, quarantine, and prompt treatment.

Efforts to curb the spread of COVID-19, in which more than 170 countries are currently fighting and controlling the disease, are ongoing, with daily statistics on the number of deaths, which is based on a kind of global alliance among all countries of the world to prevent and stop the spread of this virus. With the spread of this virus and its epidemic worldwide, the diagnosis of this disease has become a priority for the medical system of the world and international organizations such as WHO. There are currently several ways to diagnose this disease. One of the important parameters in this regard is the use of advanced equipment and the help of technology to control this virus. Artificial intelligence and machine learning techniques play a significant role in carrying out this mission.

Recently, the analysis of disease-related data, data preparation, prevention, and control of infectious diseases, such as COVID-19, has become one of the goals of artificial intelligence. Artificial intelligence is one of the technologies that can easily track the spread of the virus, identify high-risk patients, and help control infection in a timely manner. It can also predict patient mortality risk by analyzing previous data. Artificial intelligence can help us fight the virus with population screening, medical help, information, and suggestions for infection control. This technology has the potential to improve the planning, treatment, and reported outcomes of the COVID-19 patient and is an evidence-based medical tool.

Artificial intelligence can quickly analyze the symptoms and alert patients and treatment staff. This technology helps make decisions faster, which is cost-effective. Artificial intelligence helps create a new COVID-19 patient diagnosis and management system through efficient algorithms. Artificial intelligence uses medical imaging technologies such as X-ray imaging, Computed tomography (CT), and magnetic resonance imaging (MRI) to diagnose infected cases. At the same time, in the field of medical imaging, machine learning helps to identify patterns in images and enhances the ability of radiologists to diagnose and detect disease early.

The diagnosis of COVID-19 is problematic due to the appearance of different types of coronaviruses. However, sampling offers well diagnosis, it is possible only by surgery, which gives an unpleasant experience to the patient. For avoiding redundant sampling, researchers have reviewed numerous noninvasive techniques for diagnosing COVID-19. Almost, all diagnosis systems based on image processing include three main parts of image preprocessing, boundary identification, feature extraction, and the final classification [1]. However, COVID-19 is a new disease, because of its highly dangerous and pandemic status, different works have been done in the diagnosis and purpose of this cancer from medical images.

Song et al. [2] proposed diagnosis method based on CT images. They collected chest CT scans from hospitals of two provinces in China. Deep learning was used for the diagnosis of COVID-19. The final results indicated that the proposed method with 0.96 precision has good accuracy for detecting the COVID-19 patients. The method was also provided a model to extract significant lesion features from the CT images.

Zhang et al. [3] proposed deep anomaly detection system to provide a fast and reliable screening. For providing the model efficiency, Github, repository1, and Chest X-ray14 datasets were analyzed. Simulation results showed that the proposed method provides about 96.00% accuracy in the diagnosis of the COVID-19 cases with 96.00% sensitivity which are proper results for this purpose.

Jin et al. [4] presented another method based on medical imaging for a quick diagnosis of COVID-19 patients from CT scans. The method was based on a difficult multiclass diagnosis system based on Convolutional Neural Network (CNN) to reach the defective region. Moreover, the diagnosis accuracy of chest X-ray (CXR) was compared with that of CT to show its higher accuracy.

As mentioned above, X-ray imaging provides better results for diagnosing the COVID-19 disease. Therefore, in this study, we propose a medical imaging system based on X-ray to provide better results of the diagnosis. However, the results of the researches in the literature are well, but there are also lots of works that can be done on the system consistency and accuracy. Therefore, in this study, the following contributions are considered:

- A new CAD-based approach for optimal diagnosis of COVID-19 from chest X-ray images
- Using a new algorithm to decrease the complexity of feature extraction
- Using a new algorithm for the final classification of the images
- The new algorithm is based on a new metaheuristic called Archimedes optimization algorithm (AOA)
- Validating the method by three different datasets and comparing with four other state-of-the-art methods

The next sections of this paper are organized as follows. In Section 2, the main preprocessing stages of the paper, including min-max normalization and histogram equalization, are explained.  Section 3 explains about feature extraction and the features that are utilized for the classification.  In Section 4, the theory of the Archimedes optimization algorithm has been explained.  Section 5 describes the method of classification of the data based on optimization and multilayer perceptron.  In Section 6, the simulation results have been completely performed and discussion proved the method capability. Finally, the paper has been concluded in Section 7.

## 2. Preprocessing of the CXR Images

### 2.1. Min-Max Normalization

Data normalization is one of the most important stages of preprocessing in data mining science. In explaining the importance of normalization, imagine that the intervals corresponding to the values of the two properties are significantly different from each other. For example, suppose the interval for one of the attributes is the interval [1, 0] and the interval for another attribute of the same data set is [500, 1], in which case it is clear that when using criteria that are based on distance *A* feature with a smaller range will have virtually no significant effect on the calculations. According to these explanations, to achieve more accurate results, it is necessary that the intervals related to the different features be identical or close to each other. Normalization methods are used for this purpose. There are various methods for normalization that are used in different studies. In this study, the Min-Max method has been used.

In this simple method, each set of data is mapped to arbitrary intervals, the minimum and maximum values of which are already known. In this method, any desired interval can be mapped to a new interval with just a simple conversion. Suppose attribute *A* is to be mapped from the data set between min_*A*_ to max_*A*_ and the new range new_Min_ to new_Max_. For this purpose, any initial value such as *v* in the initial interval will be converted to the new value *v*′ in the new interval according to the following equation:

(1) $$\begin{array}{c} v^{\prime }=\left(v-\min_{A}\right)\times \frac{{\text{New}}_{\text{Max}}-{\text{New}}_{\text{Min}}}{\max A-\min A}+\left({\text{New}}_{\text{Min}}\right). \end{array}$$

### 2.2. Histogram Equalization

Image histogram equalization is a process that involves changes in the pixel intensity of the input image, so that the output image looks better intuitively and perceptually. Therefore, the purpose of image enhancement is to improve the interpretation or perception of the information contained therein for the viewer, or to provide better input for automated processing systems. One of the important quality factors in processing different images is contrast. If the contrast of an image is too dark, too bright, or too focused, the image information is lost in areas that are over and evenly focused. Therefore, the contrast of the image should be enhanced to show all information in the input image. The general histogram equalizer in almost all types of images is due to its simplicity and relatively good performance. The main idea of modifying the histogram is to reprogram the gray surfaces of the input image based on the uniform expansion of its probability density function. This technique flattens the dynamic range of the image histogram, increasing the contrast of the input image as much as possible.

By considering a discrete grayscale image, *x* with *n*_*i*_ as the number of occurrences of the *i*^th^ gray level, the probability of an occurrence of a pixel of the level *i* in an image is as follows:

(2) $$\begin{array}{c} v^{\prime }=\left(v-\min_{A}\right)\times \frac{{\text{New}}_{\text{Max}}-{\text{New}}_{\text{Min}}}{\max A-\min A}+\left({\text{New}}_{\text{Min}}\right), \end{array}$$

where *L* describes the total number of gray levels in an image (typically 256), *n* signifies the image total number of pixels, and *p*_*x*_(*i*) determines the histogram of the image for pixel value *i*, normalized to [0, 1]. By considering the cumulative distribution function based on *p*_*x*_, we have

(3) $$\begin{array}{c} {\text{CDF}}_{x}\left(N\right)=\sum_{i=0}^{N}p_{x},\;x=i. \end{array}$$

That shows the accumulated normalized histogram of the image.

The idea is to generate a transformation of the form *y*=*T*(*x*) to provide a new image (*y*), with a flat histogram. The generated image is a linearized cumulative distribution function (CDF) across the value range for some constant *K* is as follows:

(4) $$\begin{array}{c} {\text{CDF}}_{y}\left(N\right)=N\times K. \end{array}$$

The CDF properties let us establish such a transform as follows:

(5) $$\begin{array}{c} {\text{CDF}}_{y}\left(y^{\prime }\right)={\text{CDF}}_{y}\left(T\left(k\right)\right)={\text{CDF}}_{x}\left(k\right), \end{array}$$

where *k* is limited in the range between 0 and *L*. Notice that *T* maps the levels into the range [0, 1]; subsequently, a normalized histogram of *x* has been employed. To map the values back into the original range, the following simple transformation should be performed:

(6) $$\begin{array}{c} y^{\prime }=y\times \left(\max x-\min x\right)+\min x. \end{array}$$

More details can be derived in [5].  Figure 1 shows some examples of the image preprocessing step.

## 3. Feature Extraction

The purpose of feature extraction is to make the raw data more usable for future statistical processing. Feature extraction is a widespread process in various types of data processing such as image processing, audio processing, etc. Feature extraction means selecting a feature that can describe the image with little information. These features must have properties so that a set of these features for each image is described uniquely. Therefore, feature extraction is a process in which data is mapped from a high-dimensional space to a lower-dimensional space. This mapping can be linear (like the principal component analysis method) or nonlinear. How to select these features requires the study of data properties, and to extract it, preprocessing operations and filters must be applied to the image to turn the image into the desired information.

Numerous features are introduced for image feature extraction. In this research, geometric features, statistical features, and texture features have been employed. In the following, the formulation of this feature is explained as follows:

(7a) $$\begin{array}{c} \text{perimeter}=\sum_{I=1}^{M}\sum_{j=1}^{N}B_{p}\left(i,j\right), \end{array}$$

(7b) $$\begin{array}{c} \text{correlation}=\sum_{i=1}^{M}\sum_{j=1}^{N}\frac{p\left(i,j\right)-\mu_{r}\mu_{c}}{\sigma_{r}\sigma_{c}}, \end{array}$$

(7c) $$\begin{array}{c} \text{area}=\sum_{i=1}^{M}\sum_{j=1}^{N}p\left(i,j\right), \end{array}$$

(7d) $$\begin{array}{c} \text{solidity}=\frac{\text{area}}{\text{convex area}}, \end{array}$$

(7e) $$\begin{array}{c} \text{elongation}=\frac{2\sqrt{\text{area}}}{a\sqrt{\pi }}, \end{array}$$

(7f) $$\begin{array}{c} \text{rectangularity}=\frac{\text{area}}{b\times a}, \end{array}$$

(7g) $$\begin{array}{c} \text{irregularity index}=4\pi \times \frac{\text{area}}{{\text{perimeter}}^{2}}, \end{array}$$

(7h) $$\begin{array}{c} \text{eccentricity}=2a^{-1}{\left(a^{2}-b^{2}\right)}^{0.5}, \end{array}$$

(7i) $$\begin{array}{c} \text{form factor}=\frac{\text{area}}{a^{2}}, \end{array}$$

(7j) $$\begin{array}{c} \text{contrast}=\sum_{i=1}^{M}\sum_{j=1}^{N}p^{2}\left(i,j\right), \end{array}$$

(7k) $$\begin{array}{c} \text{mean}=\frac{1}{MN}\sum_{i=1}^{M}\sum_{j=1}^{N}p\left(i,j\right), \end{array}$$

(7l) $$\begin{array}{c} \text{entropy}=-\sum_{i=1}^{M}\sum_{j=1}^{N}p\left(i,j\right)\log\;p\left(i,j\right), \end{array}$$

(7m) $$\begin{array}{c} \text{variance}=\frac{1}{MN}\sum_{i=1}^{M}\sum_{j=1}^{N}\left(p\left(i,j\right)-\mu \right), \end{array}$$

(7n) $$\begin{array}{c} \text{standard deviation}={\text{variance}}^{\left(1/2\right)}, \end{array}$$

(7o) $$\begin{array}{c} \text{energy}=\sum_{i=1}^{M}\sum_{j=1}^{N}p^{2}\left(i,j\right), \end{array}$$

(7p) $$\begin{array}{c} \text{homogenity}=\sum_{i=1}^{M}\sum_{j=1}^{N}\frac{p\left(i,j\right)}{1+\left|i-j\right|}. \end{array}$$

Invariant moments:

(7q) $$\begin{array}{c} \varphi_{1}=\eta_{20}+\eta_{02},\\ \varphi_{2}={\left(\eta_{20}-\eta_{02}\right)}^{2}+4\eta_{11}^{2},\\ \varphi_{3}={\left(\eta_{30}-3\eta_{12}\right)}^{2}+{\left(3\eta_{21}-\mu_{03}\right)}^{2}, \end{array}$$

where *MN* defines the image size, *B*_*p*_ signifies the length of the external side for the boundary pixel, *p*(*i*, *j*) states the value of the intensity of the pixel at location (*i*,  *j*), *a* defines the major axis, and *b* determines the minor axis, *μ* signifies the mean value *σ* describes the standard deviation.

Yet, some of the explained features have a low effect and some others have a high effect on the diagnosis of the image. In this study, an optimized procedure is utilized for a better selection of the useful features from the image. Therefore, in this study, we consider the important features selection as an optimization problem. The objective function is formulated as follows:

(8) $$\begin{array}{c} \text{fitness}=\frac{\left(\text{TP}\times \text{TN}\right)-\left(\text{FP}\times \text{FN}\right)}{\sqrt{\left(\left(\text{TN}+\text{FP}\right)\times \left(\text{TP}+\text{FP}\right)\times \left(\text{TP}+\text{FN}\right)\times \left(\text{TN}+\text{FN}\right)\right)}}, \end{array}$$

where FP, FN, TP, and TN represent false positive, false negative, true positive (TP), and true negative (TN).

To get the best value of this problem, we need a proper optimizer. Different kinds of optimization methods can be used for this, but due to the complexity and nonlinear behavior of this study, it is better to use a metaheuristic. The present study uses Archimedes optimization algorithm as one of the newest and efficient metaheuristics to solve this problem. More explanation about this algorithm is given in the next section.

## 4. Archimedes Optimization Algorithm

The goal of optimization is to find the best acceptable solution, given the limitations and needs of the problem. For a problem, there may be different solutions, and to compare them and to select the optimal solution, a function called the objective function is defined. The choice of this function depends on the nature of the problem. The purpose of optimization is to determine the design variables so that the objective function is minimized or maximized.

There are different types of optimization methods. In the meantime, heuristic algorithms provide good results rather than classical methods in solving optimization problems. The purpose of heuristic algorithms is to provide a solution within an acceptable time frame that is appropriate to solve the problem. The heuristic algorithm may not be the best real solution to the problem, but it can be close to the best solution.

The heuristic algorithms can be combined with optimization algorithms to improve the performance of the algorithm. A metaheuristic algorithm combines heuristic algorithms designed to find, generate, or select any exploration at any stage and provides a good solution to problems that have optimization problems. Metaheuristic algorithms take into account some of the optimization assumptions that need to be solved.

Metaheuristic algorithms are techniques that are inspired by nature, physics, and human beings and are used to solve many optimization problems. Usually, metaheuristic algorithms are used in combination with other algorithms to achieve the optimal solution or to exit the local optimal solution status. In recent years, one of the most important and promising researches has been “heuristic methods taken from nature.” These methods have similarities with social or natural systems.

Their application is derived from continuous metaheuristic methods that have had very good results in solving problem problems (NP-Hard). Based on the no-free-lunch theorem, each metaheuristic algorithm has some advantages and disadvantages. Therefore, an algorithm may have the best results for a specific problem, while it gives the worst results on another problem.

This motivation makes the researchers work on different new metaheuristics to provide the better one continuously. For example, Variance Reduction of Gaussian Distribution (VRGD) [6, 7], Chimp Optimization Algorithm (COA) [8], World Cup Optimization (WCO) Algorithm [9], Red Fox Optimization (RFO) algorithm [10], Equilibrium optimizer [11], and Archimedes optimization algorithm [12] are some of the newly introduced metaheuristic algorithms.

Among the mentioned algorithms, the Archimedes optimization is the most newly introduced population-based metaheuristic algorithm, which is inspired by the Archimedes' principle and the buoyancy law. This principle simulates the time an object is immersed partially or fully in fluid, the fluid employs an upward force on the object, which is equal to the fluid discharged weight by the object.

The Archimedes optimizer is an algorithm based on a population with consideration of the immersed objects as candidates. AOA starts with several random numbers being distributed consistently with a possible limitation, similar to other metaheuristics based on the population. The searching method of objects includes random volumes (*V*), densities (*D*), and accelerations (*A*). The Archimedes optimizer can be introduced as a global optimization method by consideration of exploitation and exploration. This technique is described in the following. The initialization of the location of candidates is a phased one as defined below:

(9) $$\begin{array}{c} x\left(i\right)=x_{l}\left(i\right)+\text{rand}\times \left(x_{u}\left(i\right)-x_{l}\left(i\right)\right),\;i=1,2,\ldots ,N, \end{array}$$

where *x*(*i*) is the *i*^th^ candidate with *N* candidates in a population and *x*_*l*_(*i*) and *x*_*u*_(*i*) stand for the minimum and maximum ranges of the solution space.

As aforementioned, *V*, *D*, and *A* are initialized randomly for each *candidate* by this algorithm.

The update of *V*, *D*, and *A* for the *i*^th^ candidate for the iteration *t*+ is phase two as follows:

(10) $$\begin{array}{c} V\left(i\right)=\text{rand},\\ D\left(i\right)=\text{rand},\\ A\left(i\right)=x_{l}\left(i\right)+\text{rand}\times \left(x_{u}\left(i\right)-x_{l}\left(i\right)\right). \end{array}$$

This algorithm computes the primary individuals and the candidates with optimum cost numbers are chosen here. These optimum amounts have been specified as *V*^best^, *D*^best^, *A*^best^, and *x*^best^.

Then, by the algorithm parameters, the objects have been updated. By the collision condition of the acceleration of the object with neighborhood objects, they are updated. Next, *V*, *D*, and *A* parameters are used to achieve the updated locations of the candidates. This is defined as follows:

(11) $$\begin{array}{c} V^{t+1}\left(i\right)=V^{t}\left(i\right)+\text{rand}\times \left(V^{\text{best}}-V^{t}\left(i\right)\right),\\ D^{t+1}\left(i\right)=D^{t}\left(i\right)+\text{rand}\times \left(D^{\text{best}}-D^{t}\left(i\right)\right), \end{array}$$

where *V*^best^ and *D*^best^ signify the volume and the density of the optimum candidate, and rand defines a consistent randomly distributed number.

The application of a transfer operator (TF) and *D* factor is to transfer from exploration to exploitation. This is obtained as follows:

(12) $$\begin{array}{c} \text{TF}=\exp\left(\frac{t-t^{\max}}{t^{\max}}\right), \end{array}$$

where TF is stepped up gradually in duration to reach 1, *t* is the number of iterations, and *t*^max^ is the highest number of iterations. Consequently, a reduction factor of *D* tries the algorithm to obtain a global to local search, which is defined as follows:

(13) $$\begin{array}{c} D^{t+1}=\exp\left(\frac{t^{\max}-t}{t^{\max}}\right)-\;\left(\frac{t}{t^{\max}}\right), \end{array}$$

where *D*^*t*+1^ minimizes slowly to give a suitable convergence. Thus, the balance between exploitation and exploration is possible by this.

If TF ≤ 0.5, candidates are considered without collision for exploitation, and the acceleration of the candidate is updated by the algorithm for *i*+1 iteration as defined below:

(14) $$\begin{array}{c} D^{t+1}=\exp\left(\frac{t^{\max}-t}{t^{\max}}\right)-\;\left(\frac{t}{t^{\max}}\right), \end{array}$$

where *D*^*t*+1^ decreases over time which can converge in the former found promising area.

This leads to a proper balance between exploration and exploitation in the AOA algorithm. Then, to update the candidate acceleration for iteration *t*+1, a random material (mr) was chosen as follows:

(15) $$\begin{array}{c} A^{t+1}=\frac{D_{\text{mr}}+V_{\text{mr}}\times A_{\text{mr}}}{D^{t+1}\left(i\right)\times V^{t+1}\left(i\right)}, \end{array}$$

where *A*(*i*), *V*(*i*), and *D*(*i*) denote the acceleration, volume, and density of the *i*^th^ candidate, respectively, while *A*_mr_, *D*_mr_, and *V*_mr_ define the acceleration, volume, and density of random material (mr). Exploration-exploitation performance can be altered by a performance value different from 0.5.

The exploitation of the algorithm was modeled without any collision between the candidate if TF > 0.5. The update of the candidates was performed as below in this step:

(16) $$\begin{array}{c} A^{t+1}\left(i\right)=\frac{D^{\text{best}}+V^{\text{best}}\times A^{\text{best}}}{D^{t+1}\left(i\right)\times V^{t+1}\left(i\right)}, \end{array}$$

where the optimum candidate acceleration is specified by *A*^best^.

Therefore, the normalized acceleration can be obtained as follows:

(17) $$\begin{array}{c} A^{t+1}\left(\bar{i}\right)=u\times \frac{A^{t+1}\left(i\right)-\min\left(A\right)}{\max\left(A\right)-\min\left(A\right)}+l, \end{array}$$

where *A*^*t*+1^(*i*) defines the step variation percentage of each population and *l* and *u* explain the normalization restriction between 0.9 and 0.1, respectively.

In the later phase, the location of the *i*^th^ updated candidate for iteration *t*+1 if TF ≤ 0.5 was obtained as follows:

(18) $$\begin{array}{c} x^{t+1}\left(i\right)=x^{t}\left(i\right)+c_{1}\times \text{rand}\times A^{t+1}\left(\bar{i}\right)\times D\times \left(x^{\text{rand}}-x^{t}\left(i\right)\right), \end{array}$$

where *C*_1_ denotes a constant equal to 2.

Otherwise, the candidates renew their locations if TF > 0.5  as follows:

(19) $$\begin{array}{c} x^{t+1}\left(i\right)=x^{{\text{best}}^{t}}+F\times c_{2}\times \text{rand}\times A^{t+1}\left(\bar{i}\right)\times D\times \left(T\times x^{\text{best}}-x^{t}\left(i\right)\right), \end{array}$$

where *T* increments over time between *c*_3_ × 0.3 and 1 and considers a defined percentage of the optimum location and *c*_2_ denotes a constant amount of 6. This amount increases over time to decrease the difference between the present and the optimum locations to give a proper balance between exploration and exploitation, and *F* states the updated model of the candidates by their locations, which is defined as follows:

(20) $$\begin{array}{c} F=\left\{\begin{array}{cc} +1, & \text{if }P\leq 0.5,\\ +1, & \text{if }P>0.5, \end{array}\right. \end{array}$$

where

(21) $$\begin{array}{c} P=2\times \text{rand}-c_{4}. \end{array}$$

The AOA evaluates each candidate by fitness function *f* and saves the optimum solution. The application of AOA here is to minimize Fitness function that is described in the previous section.

## 5. Image Classification

To provide a proper classification, the CXR images are grouped into two target classes where each contains 140 images including normal and COVID-19. Here, an optimized multilayer neural network (MLP) has been utilized. In this research, the proposed AOA is used again to design an optimal classifier based on MLP neural network. The main purpose here is to optimize the value of the weight to accomplish an MLP with global optimal.

Generally, artificial neural networks (ANNs) are computing systems inspired by biological neural networks. These systems learn activities by looking at examples (i.e., they improve their performance by performing activities over time), and this usually happens without any activity-specific programming. An ANN is based on a set of connected units or nodes, called artificial neurons (similar to biological neurons in the animal brain). Any connection (synapse) between neurons can transmit a signal from one neuron to another. The receiving neuron (postsynaptic) can process the signal (*s*) and then the signal neurons attached to it. In typical ANN implementations, a synapse signal is a real number, and the output of each neuron is calculated by a nonlinear function of its inputs. Neurons and synapses usually have weights that are adjusted as learning progresses. This weight increases or decreases the signal strength it sends to the synapse. Neurons can have a threshold at which a signal can only be sent if the total signal is absorbed by that threshold.

One of the most basic neural models available is the multilayer perceptron (MLP) model, which simulates the transfer function of the human brain. In this type of neural network, most of the behaviors of human brain networks and signal propagation have been considered, and hence, they are sometimes referred to as feedforward networks. Each neuron in the human brain, called a neuron, processes the input (from another neuron or nonneuron) and transmits the result to another cell (neuron or nonneuron). This behavior continues until a definite result is reached, which is likely to eventually lead to a decision process, thought, or move. Widely used supervision in neural networks is backpropagation, which is based on the error correction law. Assume a neural network output as *y*. This function is reliant on the inputs, *x*_*i*_, and their weights.

(22) $$\begin{array}{c} y\left(t\right)=f\left(\sum_{i}\omega_{i}x_{i}\right), \end{array}$$

where *α* signifies the activation function (here the sigmoid function has been used).

Backpropagation is a classic method based on gradient descent to adjust the network weights such that network errors get minimized. This technique takes a lot of time.

One big issue in using gradient descent algorithms is that they are sometimes stuck in the local minimum which is reliant on the initial weight. Therefore, they need a global minimizer for refining this issue. This leads us to use again AOA, this time for classification of the COVID-19 data.

The main purpose of AOA here is to adjust the network weights such that the network mean squared error (MSE) between the experimental data and the network value get minimized; that is,

(23) $$\begin{array}{c} \min\text{ MSE}=\frac{1}{2}\sum_{k=1}^{n}\overset{m}{\underset{j=1}{\sum }}{\left(Y_{j}-T_{j}\right)}^{2}, \end{array}$$

where *m* states the number of output nodes, *n* signifies the number of training samples, and *Y*_*j*_ and *T*_*j*_ represent the real output and the desired output, respectively.

## 6. Simulation Results

### 6.1. The Database

Recently, some different datasets have been introduced for COVID-19. This research adopts reliable resources provided by the Renmin Hospital of Wuhan University and two affiliated hospitals (the Third Affiliated Hospital and Sun Yat-sen Memorial Hospital) of the Sun Yat-sen University in Guangzhou with 76 and 12 patients, respectively [13].  Figure 2 shows some examples of the utilized dataset for the COVID-19.

### 6.2. System Configuration

In this study, we used an optimized X-ray diagnosis system for COVID-19 disease detection.  Figure 3 shows the graphical abstract of the proposed system. As can be observed from Figure 3, the proposed CAD-based COVID-19 X-ray diagnosis system has four main steps. First, the input image has been preprocessed based on min-max normalization to scale all data into a normal scale, and the scaled images have been improved based on the histogram equalization. Then, geometric features, statistical features, and texture features are extracted from the images. In the next step, the useless or less informative features have been removed to increase the system speed, and the final step is the classification of the features based on an optimized MLP network.

As previously mentioned, Archimedes optimization algorithm is used to adjust the weights and train the proposed multilayer neural network with minimum error. The main parameter setting for the network is reported in Table 1.

The experiment has been established on MATLAB R2016b 64-bit version and executed on computation environment of Intel® Pentium® CPU 2.30 GHz, 2.3 GHz, 4 GB RAM, and 64-bit Windows 7 operating system. The training stage has been iterated 15 times independently to obtain reliable results. During the training of the proposed model, both training and validation sets were reached.  Figure 4 shows the loss graph of the model.

As can be observed from the loss graph in Figure 4, there is a satisfying fit between the validation and the training curves that confirms the suggested model's efficiency and with no further overfitting or underfitting. The analysis has been accomplished based on five performance indexes including accuracy, specificity, precision, recall, and *F*1-score that are formulated follows:

(24a) $$\begin{array}{c} \text{accuracy}=\frac{\text{TP}+\text{TN}}{\text{TP}+\text{FP}+\text{TN}+\text{FN}}, \end{array}$$

(24b) $$\begin{array}{c} \text{specificity}=\frac{\text{TN}}{\text{TN}+\text{FN}}, \end{array}$$

(24c) $$\begin{array}{c} \text{precision}=\frac{\text{TP}}{\text{TP}+\text{FP}}, \end{array}$$

(24d) $$\begin{array}{c} \text{recall}=\frac{\text{TP}}{\text{TP}+\text{FN}}, \end{array}$$

(24e) $$\begin{array}{c} F_{1}-\text{score}=\frac{\text{precision}+\text{recall}}{2}, \end{array}$$

where TP, FP, TN, and FN represent the numbers of true positives, false positives, true negatives, and false negatives, respectively.

The final results are compared with four other methods including Ismail's method [14], Mangal's method [15], Abbas's method [16], and Castiglioni's method [17].  Table 2 reports the performance analysis of the proposed method compared with other state-of-the-art techniques.

As can be observed from Table 2, the proposed method achieved the highest accuracy score among all studied methods, and Ismail's and Abbas's methods are close, and Mangal's method has the lowest score. By analyzing the *F*-measurement, another balanced measurement, the proposed method has ranked and Mangal's and Abbas's methods with close values are ranked as the lowest scores, while Castiglioni's method has slightly higher than these two methods.

## 7. Conclusions

The new coronavirus, which causes COVID-19 disease, is one of the seven viruses in the coronavirus family that are transmitted from one human to another. This disease is spreading around the world and makes lots of cases and deaths every day. One of the methods for the detection of this disease is to use chest X-ray images. The present study proposed a CAD procedure for automatic diagnosis of COVID-19 from chest X-ray images. At first, the original X-ray images were preprocessed by min-max normalization to scale all data into a normal scale, and then histogram equalization was performed to improve the quality of the images before main processing. In the next step, geometric features, statistical features, and texture features were extracted from the X-ray images. Afterward, by performing an optimized method for feature selection, the useless features were removed. The optimization of feature selection and the MLP classifier was based on a newly introduced metaheuristic, called Archimedes optimization algorithm. Finally, an optimized MLP network was used to determine the suspected cases of the COVID-19. Simulations were performed in Renmin Hospital of Wuhan University and two affiliated hospitals (the Third Affiliated Hospital and Sun Yat-sen Memorial Hospital) of the Sun Yat-sen University in Guangzhou dataset, and the results were compared with four state-of-the-art methods to examine the model efficiency. Final results specified that with analyzing accuracy, specificity, precision, recall, and *F*1-score, the proposed method has the best efficiency toward the other methods. As can be inferred from the results, the proposed method provides a good optimal result for the diagnosis of COVID-19. However, in some cases, the method has weak results. This leads us to work more on developing the AOA in the future work to provide better results. The future work will be to propose a new method for improving the algorithm efficiency and to provide a method with higher speed to use in real-time applications.

## Figures and Tables

**Figure 1:** Some examples of preprocessing. (a) Original CXR images, (b) histogram of (a), (c) preprocessed images, and (d) histogram of (c).

**Figure 2:** Some examples of the utilized dataset for COVID-19.

**Figure 3:** The graphical abstract of the proposed system.

**Figure 4:** The loss graph of the model.

**Table 1:** The main parameter setting for the network.

Parameter	Value
Batch size	2
Maximum epochs	120
Training percentage	70
Validation percentage	15
Testing	15
Dropout value	0.2
Learning rate	0.001

**Table 2:** Performance analysis of the proposed method compared with other state-of-the-art techniques.

Method	Performance metric				
	Accuracy (%)	Specificity (%)	Precision (%)	Recall (%)	*F*-measure (%)
Ismail's method [14]	84	80	93	88	90.5
Mangal's method [15]	83	75	93	93	93
Abbas's method [16]	84	78	94	92	93
Castiglioni's [17]	82	79	95	93	94
Proposed method	86	79	96	96	96

## Data Availability

This research adopts reliable resources provided by the Renmin Hospital of Wuhan University and two affiliated hospitals (the Third Affiliated Hospital and Sun Yat-sen Memorial Hospital) of the Sun Yat-sen University in Guangzhou with 76 and 12 patients. The dataset can be accessed by sending a request to these hospitals.
